# Down-regulated lncRNA DLX6-AS1 inhibits tumorigenesis through STAT3 signaling pathway by suppressing CADM1 promoter methylation in liver cancer stem cells

**DOI:** 10.1186/s13046-019-1239-3

**Published:** 2019-06-06

**Authors:** Dong-Mei Wu, Zi-Hui Zheng, Ying-Bo Zhang, Shao-Hua Fan, Zi-Feng Zhang, Yong-Jian Wang, Yuan-Lin Zheng, Jun Lu

**Affiliations:** 1 Key Laboratory for Biotechnology on Medicinal Plants of Jiangsu Province, School of Life Science, Jiangsu Normal University, Xuzhou, 221116 Jiangsu Province People’s Republic of China; 2 College of Health Sciences, Jiangsu Normal University, Xuzhou, 221116 Jiangsu Province People’s Republic of China; 3 State Key Laboratory Cultivation Base For TCM Quality and Efficacy, School of Medicine and Life Sciences, Nanjing University of Chinese Medicine, Nanjing, 210023 People’s Republic of China; 4 Department of Pathology, Qiqihar Medical University, Qiqihar, 161006 People’s Republic of China

**Keywords:** LncRNA DLX6-AS1, CADM1, STAT3 signaling pathway, Hepatocellular carcinoma, Liver cancer stem cell

## Abstract

**Background:**

Liver cancer stem cells (LCSCs) are a small subset of cells characterized by unlimited self-renewal, cell differentiation, and uncontrollable cellular growth. LCSCs are also resistant to conventional therapies and are thus believed to be held responsible for causing treatment failure of hepatocellular carcinoma (HCC). It has been recently found that long non-coding RNAs (lncRNAs) are important regulators in HCC. This present study aims to explore the underlying mechanism of how lncRNA DLX6-AS1 influences the development of LCSCs and HCC.

**Methods:**

A microarray-based analysis was performed to initially screen differentially expressed lncRNAs associated with HCC. We then analyzed the lncRNA DLX6-AS1 levels as well as CADM1 promoter methylation. The mRNA and protein expression of CADM1, STAT3, CD133, CD13, OCT-4, SOX2, and Nanog were then detected. We quantified our results by evaluating the spheroid formation, proliferation, and tumor formation abilities, as well as the proportion of tumor stem cells, and the recruitment of DNA methyltransferase (DNMT) in LCSCs when lncRNA DLX6-AS1 was either overexpressed or silenced.

**Results:**

LncRNA DLX6-AS1 was upregulated in HCC. The silencing of lncRNA DLX6-AS1 was shown to reduce and inhibit spheroid formation, colony formation, proliferation, and tumor formation abilities, as well as attenuate CD133, CD13, OCT-4, SOX2, and Nanog expression in LCSCs. Furthermore, downregulation of lncRNA DLX6-AS1 contributed to a reduction in CADM1 promoter methylation via suppression of DNMT1, DNMT3a, and DNMT3b in LCSCs and inactivating the STAT3 signaling pathway.

**Conclusion:**

This study demonstrated that down-regulated lncRNA DLX6-AS1 may inhibit the stem cell properties of LCSCs through upregulation of CADM1 by suppressing the methylation of the CADM1 promoter and inactivation of the STAT3 signaling pathway.

**Electronic supplementary material:**

The online version of this article (10.1186/s13046-019-1239-3) contains supplementary material, which is available to authorized users.

## Background

Hepatocellular carcinoma (HCC) is the most common type of primary liver cancer. This form of malignancy ranks sixth as the most occurring cancer globally and is the third leading cause of death [1, 2]. In general, the incidence of HCC occurs higher in men than that in women worldwide [3]. Despite early detection, patients diagnosed with HCC usually have a poor prognosis which is mainly due to unobvious pathognomonic symptoms and occult onset [2]. Although surgical resection, including liver transplantation has therapeutic effects in treating patients with HCC, the prognosis of HCC still remains poor mostly due to the inhomogeneity of primary tumors, and tumor relapse [4]. Despite the widely-used use of combination chemotherapy, these approaches still fail to improve the overall survival (OS) of HCC patients [5]. HCC has been found to be caused and linked to various factors, such as autoimmune hepatitis, alcohol abuse, chronic hepatitis B/C virus infections (HBV/HCV), and some other metabolic diseases [6]. The advanced genetic technology makes it clear that many more factors than what was previously thought are revealed to be implicated in the development of HCC; however, the specific mechanism still remains elusive. According to the theory proposed by Reya et al., only a small number of cells in tumor tissue, named cancer stem cells (CSCs), have the ability for indefinite self-renewal and have the multidirectional differentiation potential to generate the heterogeneity of tumor cells [7]. Liver CSCs (LCSCs) have been regarded as the cells with specific stem cell-like features in the HCC, in which therapeutic approach is to realize specific target and eradication of LCSCs [8]. It has been indicated that long non-coding RNA (lncRNAs) may play important roles in the regulation of the biological functions of LCSCs [9].

LncRNAs refer to a class of transcripts coded in non-proteins with a length of over 200 nucleotides. LncRNAs and have been reported to be closely involved in both development and progression of a variety of tumors [10]. LncRNA distal-less homeobox 6 antisense 1 (DLX6-AS1) are regulatory of members in the DLX gene family [11]. Overexpression of DLX6-AS1 has been previously revealed in HCC tissues, which highly suggests that DLX6-AS1 could serve as an oncogene of HCC by acting via the DLX6-AS1/miR-203a/MMP-2 pathway [12]. Interestingly, DLX6-AS1 was reported to enhance osteosarcoma stemness through regulation of miR-129-5p/DLK1, suggested that DLX6-AS1 might correlate with cancer stemness [13]. In addition, cell adhesion molecule 1 (CADM1), whose expression has been extensively found in lung, brain, testis, liver, and some cancer cells [14], has been observed to be downregulated in HCC cells, serving as a propellant of tumorigenesis of HCC [15]. Research has provided evidence that HCC is more likely to recur in patients with extensive CADM1 methylation compared to patients with less or without CADM1 methylation [16]. Additionally, the signal transducer and activator of transcription 3 (STAT3)/Nanog signaling pathway have been suggested to participate in the induction of liver cancer stem cell (LCSC) properties [17]. In a recent study, CADM1 was shown to suppress STAT3 in patients with squamous cell carcinomas (SqCC) [18]. Another study also found that another type of lncRNA known as SNHG16 could regulate the STAT3 signaling pathway in carcinogenesis of HCC [19]. However, the relationship among lncRNA DLX6-AS1, CADM1 methylation, STAT3 signaling pathway remains to be investigated. Therefore, we aim to investigate whether the STAT3 signaling pathway participates in the progression of LCSCs with the hypothesis that lncRNA DLX6-AS1 could influence LCSC progression via regulation of CADM1 promoter methylation and STAT3 signaling pathway.

## Materials and methods

### Ethics statement

The study was approved by the Ethics Committee of the Affiliated Municipal Hospital of Xuzhou. All participants have signed written informed consent forms prior to the experiment. Efforts were made to relieve the mice pain as much as possible.

### Microarray-based data analysis

The Cancer Genome Atlas (TCGA) database (http://cancergenome.nih.gov/) was employed to retrieve the data of expressed genes related to HCC. The expression of DLX6-AS1 in HCC was analyzed by R language software. The transcriptome profiling data was analyzed by differential analysis with package edgeR of R [20]. The obtained *p*-value was corrected by false positive discovery (FDR) correction with package multitest. FDR < 0.05 and |log2 (fold change)| > 1 were considered as the screening criteria for differentially expressed genes (DEGs). The prediction of co-expression gene of the differentially expressed lncRNA was conducted on The Multi Experiment Matrix (MEM, http://biit.cs.ut.ee/mem/) website, and the IncATLAS (http://lncatlas.crg.eu/) was used for subcellular localization of target lncRNA. Co-expressed genes retrieved from the Kyoto Encyclopedia of Genes and Genomes (KEGG) was analyzed using the webgestal database (http://www.webgestalt.org/option.php) to confirm the co-expressed genes. The Blast results showed the existence of binding sites of DLX6-AS1 on CADM1 gene promoter region.

### Cell and tissue collection

Five HCC cell lines of SMMC-7721, HCCLM3, Hep3B, HepG2 and Huh7 and an immortalized normal L02 liver cell line were purchased from the Shanghai Institute of Biochemistry and Cell Biology of Chinese Academy of Sciences (Shanghai, China). We collected 48 primary HCC tissue samples from patients who underwent HCC surgical resection in the Affiliated Municipal Hospital of Xuzhou. Amongst the 48 patients, 36 were males and 12 were females with a mean age of 48.9 ± 4.57 years old. The survival time of patients was evaluated by the Kaplan-Meier method after a follow-up period of 60 months. During the follow-up period, the time of death was designated as the endpoint. If patients died before the end of the follow-up, the time of the last follow-up was regarded as the endpoint. The interval between the date of surgery and the time of death was defined as the OS. HCC tissues were collected in strict accordance with the specifications for specimen collection. One portion of the specimens was frozen at − 80 °C, and the other part was fixed in 10% formalin, dehydrated using an automatic dehydrator, and embedded in paraffin.

### Sorting and collection of LCSCs

HCC cells in the logarithmic growth stage were re-suspended in PBS, and incubated with 100 μL FcR-blocking reagent at a cell density of 1 × 10^7^ cells/100 μL in order to block nonspecific binding. The cells were then mixed with 100 μL of CD133 and CD13 antibodies, and incubated at 4 °C in the dark for 30 min. After centrifugation at 300×g for 10 min, cells were re-suspended to create a single cell suspension using buffer solution, sorted by flow cytometry, and collected.

### Cell grouping and treatment

The LCSCs in the logarithmic growth stage were assigned into the following eight experimental groups according to what they were treated with: blank group (cells without treatment), negative control (NC) group (cells transfected with empty plasmids), oeLncRNA DLX6-AS1 group (cells transfected with lncRNA DLX6-AS1 plasmids), shLncRNA DLX6-AS1 group (cells transfected with lncRNA DLX6-AS1 interference plasmids), shCADM1 group (cells transfected with CADM1 interference plasmids), oeLncRNA DLX6-AS1 + shCADM1 group (cells co-transfected with lncRNA DLX6-AS1 plasmids and CADM1 interference plasmids), S3I-201 group (cells treated with 100 μM STAT3 signaling pathway inhibitor S3I-201), and shCADM1 + S3I-201 group (cells treated with both S3I-201 and CADM1 interference plasmids).

### Reverse transcription quantitative polymerase chain reaction (RT-qPCR)

After total RNA extraction from cells and tissues by Trizol Reagent (Invitrogen, Carlsbad, CA, USA), the obtained RNA was reversely transcribed to form complementary DNA (cDNA) according to the instructions provided by the TaqMan MicroRNA Assays Reverse Transcription primer kit (4,427,975, Applied Biosystems Inc. Carlsbad, CA, USA). RT-qPCR was conducted using an ABI7500 quantitative PCR appliance using β-actin as the internal reference (Applied Biosystems Inc. Carlsbad, CA, USA). The 2^-ΔΔCt^ method was used to calculate the ratio of expression of the target gene in the experimental groups and the blank or NC groups, and the formulas were as follows: ΔΔCT = ΔCt _experimental group_ – ΔCt _blank group or NC group_, ΔCt = Ct _target gene_ – Ct _internal reference_. Each experiment was repeated three times. The primers of lncRNA DLX6-AS1, CADM1, STAT3, surface markers of LCSCs (CD133 and CD13), and relative transcriptional factors Nanog, SOX2, and OCT-4 were designed and synthesized by TaKaRa (Tokyo, Japan) (Table 1).

**Table 1:** Primer sequences for RT-qPCR

Gene	Primer sequences
LncRNA DLX6-AS1	F: 5′-AGT TTC TCT CTA GAT TGC CTT-3′
	R: 5′-ATT GAC ATG TTA GTG CCC TT-3′
CADM1	F: 5′-ATG GCG AGT GTA GTG CTG C-3’
	R: 5′-GAT CAC TGT CAC GTC TTT CGT-3′
STAT3	F: 5′-CAG CAG CTT GAC ACA CGG TA-3′
	R: 5′-AAA CAC CAA AGT GGC ATG TGA-3′
CD133	F: 5′-AGT CGG AAA CTG GCA GAT AGC-3′
	R: 5′-GGT AGT GTT GTA CTG GGC CAA T-3′
CD13	F: 5′-GAC CAA AGT AAA GCG TGG AAT CG-3′
	R: 5′-TCT CAG CGT CAC CCG GTA G-3′
Oct-4	F: 5′-CTG GGT TGA TCC TCG GAC CT-3′
	R: 5′--CCA TCG GAG TTG CTC TCC A-3′
SOX2	F: 5′-GCC GAG TGG AAA CTT TTG TCG-3′
	R: 5′-GGC AGC GTG TAC TTA TCC TTC T-3′
Nanog	F: 5′-TTT GTG GGC CTG AAG AAA ACT-3′
	R: 5′-AGG GCT GTC CTG AAT AAG CAG-3′
β-actin	F: 5′-GCT CGT CGT CGA CAA CGG CTC-3′
	R: 5′-CAA ACA TGA TCT GGG TCA TCT TCT C-3′

Note: RT-qPCR, reverse transcription quantitative polymerase chain reaction; R, reverse; F, forward; CADM1, cell adhesion molecule 1; STAT3, signal transducer and activator of transcription 3; LncRNA, long non-coding RNA, Oct-4, octamer-binding transcription factor 4; SOX2, SRY (sex determining region Y)-box 2

### Western blot analysis

The total proteins were extracted from cells using radioimmunoprecipitation (RIPA) cell lysis buffer (BB-3209, BestBio Co., Ltd., Shanghai, China), separated by sodium dodecyl sulfate-polyacrylamide gel electrophoresis (SDS-PAGE), and electrically transferred onto a polyvinylidene fluoride (PVDF) membrane. The membrane was sealed with the sealing solution for 1 h, followed by incubation at 4 °C overnight with the addition of following primary antibodies: rabbit polyclonal antibody to CD133 (1: 1000, ab198981), CD13 (1: 500, ab154116), Nanog (1: 500, ab80892), SOX2 (1: 1000, ab97959), OCT-4 (1: 1000, ab19857), rabbit monoclonal antibodies to STAT3 (1: 1000, ab68153) and p-STAT3 (1: 2000, ab76315) (Abcam Inc., Cambridge, MA, USA), and rabbit polyclonal antibody to CADM1 (1: 1000, A1892, ABclonal Biotech Co., Ltd., Cambridge, MA, USA). On the following day, the membrane was incubated with HRP conjugated goat anti-rabbit immunoglobulin G (IgG) (1: 5000, A21020, Abbkine, USA) at 37 °C for 1 h and developed with ECL reagent. Using glyceraldehyde-3-phosphate dehydrogenase (GAPDH) as the internal reference, the relative protein levels of target proteins were expressed as the ratio of gray value of target band to that of internal reference band. Each experiment was conducted 3 times.

### Fluorescence in situ hybridization (FISH)

The subcellular localization of lncRNA DLX6-AS1 was predicted using a bioinformatics tool (http://lncatlas.crg.eu/). FISH was carried out to confirm the subcellular localization of lncRNA DLX6-AS1 in LCSCs. According to the instructions provided by the Ribo™ lncRNA FISH probeMix (RiboBio company, Guangzhou, China), Huh7 cells were cultured in cover glasses and transferred to 6-well plates, allowing them to incubate for one day in order let the cell confluence reach approximately 80%. Next, cells were fixed in 1 mL 4% paraformaldehyde at room temperature, followed by treatment with 2 μg/mL protease K, glycine, and ethyl phthalate reagent. After that, cells were incubated with 250 μL prehybridization solution at 42 °C for 1 h, and then incubated with 250 μL of 300 ng/mL hybridization solution containing probe at 42 °C overnight after removing the prehybridization solution. The cells were then washed with phosphate-buffered saline with Tween-20 (PBST), incubated with 4′,6-diamidino-2-phenylindole (DAPI) (1: 800) for five minutes in a 24-well plate, followed by a PBST rinse. Finally, cells were sealed with anti-fluorescence quenching agent. By randomly selecting give different visual fields, cells were observed and photographed under a fluorescence microscope (Olympus Optical Co., Ltd., Tokyo, Japan).

### Dual-luciferase reporter gene assay

CADM1 wild-type (WT) containing DLX6-AS1 binding sites on the CADM1 promoter region and CADM1 mutant type (MUT), were ligated into PGLO vectors respectively. Either PGLO-CADM1 WT or PGLO-CADM1-MUT was co-transfected with oeLncRNA DLX6-AS1 or NC plasmid into LCSCs. After 24 h of transfection, the cells were collected and lysed. Luciferase activity was detected using a Dual-Luciferase® Reporter Assay System (E1910, Promega, Madison, WI, USA). The relative luciferase activity was expressed as the ratio of firefly luciferase activity to renilla luciferase activity. The experiments were conducted 3 times.

### Chromatin immunoprecipitation (ChIP)

The enrichment of DNMT1, DNMT3a, and DNMT3b in the CADM1 gene promoter region was assessed using a ChIP kit (Millipore Inc., Billerica, MA, USA). After LCSCs were selected and cultured, they were incubated until cell confluence reached 70–80%. LCSCs were then obtained and fixed in 1% formaldehyde for 10 min at room temperature to crosslink DNA and protein. Cells were randomly lysed using ultrasonic treatment with 15 cycles of 10-s ultrasonic at an interval of 10 s into fragments of appropriate size. The cells were then centrifuged at 302373×g at 4 °C and the supernatant was collected. Incubation was carried out at 4 °C overnight with following specific antibodies: rabbit anti DNMT1 [ab13537], rabbit anti DNMT3a [ab2850], or rabbit anti DNMT3b [ab2851) [Abcam Inc., Cambridge, MA, USA]). Mouse IgG was used as the negative control and an antibody against RNA polymerase II was used as the positive control. The antibody bound DNA-protein compound was then precipitated with either agarose or sepharose and dissociated at 65 °C overnight. The DNA fragments were extracted and purified by hydroxybenzene or chloroform. The conjugations of CADM1 with DNMT1, DNMT3a, and DNMT3b were detected by PCR using primers specific to the CADM1 promoter region.

### RNA immunoprecipitation (RIP)

This part of the experiment was conducted in accordance with the instructions provided by the Magna RIP RNA-Binding Protein Immunoprecipitation kit (Millipore Inc., Billerica, MA, USA). LCSCs were first lysed with 100 μL cell lysis buffer containing protease inhibitor and ribonuclease inhibitor and centrifuged at 25764×g at 4 °C for 3 min. The supernatant was then collected and incubated with the corresponding 1 μg antibodies: NC antibody, IgG of normal mice, and specific antibody, rabbit antibody against target proteins (DNMT1 [ab13537], DNMT3a [ab2850], and DNMT3b [ab2851) [Abcam Inc., Cambridge, MA, USA]). After incubation with 10 to 50 μL protein A/G-beads at 4 °C overnight, and washed with 1 mL cell lysis buffer 3 to 4 times, the supernatant was then centrifuged at 179×g for 1 min at 4 °C and subjected to heat treatment with 15 μL of 2 × sodium dodecyl sulfate (SDS) for 10 min. The RNA was then extracted and RT-qPCR was performed to test the interactions DNMT1, DNMT3a, and DNMT3b with lncRNA DLX6-AS1 using the primers specific to lncRNA DLX6-AS1.

### Bisulfite sequencing PCR (BSP) and methylation-specific PCR (MSP)

Genomic DNA was extracted from LCSCs and subjected to DNA methylation using a Methyl Detector TM Bisulfite Modification Kit (Active Motif, Carlsbad, CA, USA), followed by PCR amplification. The primer sequences for CADM1 promoter were as follows: the upstream primer was 5′-GGATTTGTTTTTTTATTT-3′, and the downstream primer was 5′-AATCAAAAAAAAAATATTCTCC-3′. The reaction was conducted at 95 °C for 5 min, with 33 cycles of 95 °C for 1 min, 58 °C for 2 min and 72 °C for 1 min, and 72 °C for 10 min. In the MSP results, the appearance of the M band represented methylation (+), while the appearance of U band represented no methylation (−). In the BSP results, the data > 50% represented methylation (+), while the figure < 10% represented un-methylation (−).

### Immunofluorescence staining

The transfected LCSCs were cultured in immunofluorescence chambers with a cell density of 2 × 10^5^ cells per well. When the cell confluence reached 90%, the cells were fixed in 4% polyformaldehyde at room temperature for 15 min. After that, the cells were treated with 0.3% Triton X-100 and blocked with goat serum for 30 min. Next, cells were incubated with the STAT3 primary antibody (1: 200, ab68153, Abcam Inc., Cambridge, MA, USA) at 4 °C overnight, secondary antibody at room temperature in the dark for one hour, and DAPI solution for 15 min also in the dark. Finally, the cells were mounted with a fluorescence quenching agent and observed and photographed under a fluorescence microscope.

### Onco-spheroids formation assay

A total of 1 × 10^4^ LCSCs were seeded and distributed in a 96-well low adsorption plate and cultured with serum-free Dulbecco’s modified Eagles Medium (DMEM)-F12. They were then conjugated with 20 ng/mL epidermal growth factor (EGF) and 20 ng/mL fibroblast growth factors (FGF)-β for 10 days with semi-quantitative fluid exchange every 2 days. After 10 days, the cells were observed and counted, followed by image capture using an electron microscope.

### Soft agar colony formation (SACF) assay

One mL cell suspension was mixed with 1 mL 0.7% agarose in DMEM to obtain a cell density of 1 × 10^4^ cells/100 cm^2^ and seeded into a 100-mm-diameter container pre-covered with 0.7% agarose. Three parallel samples were set for each group. A total of 2–3 mL culture medium was added to the surface of solidified agar in a dropwise manner after which the cells were then incubated with 5% CO_2_ at 37 °C, replacing the medium every 2 to 3 days. After a month, the cells were counted under an inverted microscope, and the opaque spots with ≥ 50 cells were regarded as one colony. Images were photographed and stored for later analysis.

### 5-ethynyl-2′-deoxyuridine (EdU) staining

Cells in the logarithmic growth stage were seeded in a 96-well plate with a cell density of 4 × 10^3^–1 × 10^5^ cells per well. After seeding, cells were and cultured to normal growth phase. 50 μM EdU medium was prepared along with the cell culture medium. A total of 100 μL 50 μM EdU medium was added into each well and allowed to be incubated for 2 h. Each well was fixed with 50 μL PBS containing 4% polyformaldehyde for 30 min at room temperature followed with the addition of 50 μL 2 mg/mL glycine. The cells were left to incubate on a decolorizing rocker for 5 min. Each well was then incubated with 100 μL penetrating agent (PBS containing 0.5% Triton X-100) for 10 min. A total of 100 μL 1 X Apollo® dye solution was then added into each well, and the cells were incubated on a decolorizing rocker at room temperature in the dark for another 30 min. The cells were then washed 2 to 3 times, 10 min each time with the penetrating agent and rinsed with 100 μL methanol 1 to 2 times, 5 min each time. Next, 100 μL Hoechst33342 reaction solution was added to the cells and left to incubate in the dark at room temperature for 30 min. Finally, cells in each well were washed with 100 μL PBS 1 to 3 times.

### Limiting dilution assay (LDA) in vivo

The cells were cultured in a low-adhesion plate for 7 d, after which LCSC clumps of each group were centrifuged in a 10 mL glass centrifuge tube. The cells were washed with normal saline and detached to form single cells. Cells of different quantities (1 × 10^3^, 5 × 10^3^, 1 × 10^4^, and 5 × 10^4^) were first re-suspended in 50 μL normal saline, mixed with 50 μL Matrigel Matrix (1: 1), followed by inoculation into the subcutaneous tissue of NOD-SCID mice. Two weeks after inoculation, the formation of tumor cells was observed and recorded. The ratio of tumor stem cells to total cells was determined using the extreme limiting dilution analysis (ELDA) software (http://bioinf.wehi.edu.au/software/elda/index.html) [21].

### Tumor xenograft in NOD-SCID mice

The cells were cultured in a low-cell adhesion plate for 7 days followed by LCSC ball collection. Cells were washed with normal saline, triturated gently and prepared into a single cell suspension, followed by cell counting. A total of 2 × 10^6^ cells were re-suspended in 50 μL normal saline, mixed with 50 μL Matrigel Matrix (1: 1), and inoculated into the subcutaneous tissue of NOD-SCID mice with 8 mice in each group. Two weeks later, the volume and size of the tumor were observed and recorded.

### Statistical analysis

All the data were performed using SPSS 21.0 (IBM, Armonk, NY, USA). The measurement data were expressed as mean ± standard deviation. Differences between two groups were analyzed by *t*-test, while that among multiple groups was analyzed by one-way analysis of variance, followed by a Turkey’s post hoc-test. Values of *p* < 0.05 indicate statistical significance.

## Results

### LncRNA DLX6-AS1 is expressed at high levels in both LCSCs and HCC cells

The levels of lncRNA DLX6-AS1 in LCSCs and HCC cells were initially analyzed from the TCGA database which showed that DLX6-AS1 was overexpressed in HCC (Fig. 1a). A total of 48 HCC tissues and adjacent normal tissues were collected from HCC patients to detect the level of DLX6-AS1. According to RT-qPCR results shown in Fig. 1b & f and Additional file 1: Table S1, HCC tissues exhibited higher levels of DLX6-AS1 compared to adjacent normal tissue. This showed that the expression of DLX6-AS1 was associated with the prognosis of HCC. We measured the expression of DLX6-AS1 in some HCC cell lines (Fig. 1c) and found that the expression of DLX6-AS1 was higher in SMMC-7721, HCCLM3, Hep3B, HepG2, and Huh7 cells compared to L02 cells.

**Fig. 1:** High DLX6-AS1 expressions are observed in LCSCs and HCC cells. **a**, analysis of expression of DLX6-AS1 from TCGA database; **b**, relative expression of DLX6-AS1 in HCC tissues and adjacent normal tissues; ^*^, *p* < 0.05, vs. adjacent normal tissues; **c**, relative expression of DLX6-AS1 in immortalized normal liver cell line and HCC cell line; ^*^, *p* < 0.05, vs. the L02 cells; **d**, relative expression of DLX6-AS1 in non-spheroids and spheroids of LCSCs; ^*^, *p* < 0.05, vs. non-spheroids; **e**, relative expression of DLX6-AS1 in CD133^−^ CD13^−^ and CD133^+^ CD13^+^ HCC cells; ^*^, *p* < 0.05, vs. the CD133^−^ CD13^−^; **f**, relationship between DLX6-AS1 expression and HCC prognosis (*n* = 48); the statistical data were expressed as mean value of standard error, the differences between two groups were analyzed by *t* test, and the others were analyzed by one-way ANOVA; ANOVA, analysis of variance; *N* = 48, the experiment was conducted 3 times; LCSCs, liver cancer stem cells; LncRNA, long non-coding RNA; DLX6-AS1, DLX6 antisense RNA 1; HCC, hepatocellular carcinoma; LCSCs, liver cancer stem cells

LCSCs were enriched in low-adhesion sphere culture in order to further explore the expression of DLX6-AS1 by RT-qPCR. As shown in Fig. 1d, compared with non-sphere LCSCs, we found that the expression of DLX6-AS1 was higher in LCSC spheres. Since CD133 and CD13 were common LCSCs markers, flow cytometry was conducted to sort the cells that expressed CD133 and CD13 positive or negative cells from the Huh7 and HepG2 expressing cells. By detecting DLX6-AS1, we found that DLX6-AS1 was higher in CD133^+^ CD13^+^ positive cells compared to CD133^−^ CD13^−^ cells (Fig. 1e). These findings help demonstrate that LCSCs and HCC cells exhibited high expression of DLX6-AS1.

### Downregulation of lncRNA DLX6-AS1 suppresses self-renewal, amplification, and proliferation of LCSCs

LCSCs enriched from the Huh7 and HepG2 cells were transfected with different plasmids by low-adhesion sphere culture. The expression changes of LCSCs surface markers and transcription factors were determined using RT-qPCR and western blot analysis. In contrast to the blank and NC groups, the expression of LCSCs surface markers, CD133 and CD13, and transcription factors Nanog, SOX2, and OCT-4 were all found to elevated in the oeLncRNA DLX6-AS1 group but were all downregulated in the shLncRNA DLX6-AS1 group (Fig. 2a-c). Spheroids formation assay showed that the number of spheroids in the oeLncRNA DLX6-AS1 group was increased significantly, while that in the shLncRNA DLX6-AS1 group significantly decreased when compared with the blank and NC groups. This suggests that overexpression of DLX6-AS1 promoted the self-renewal of LCSCs (Fig. 2d). In addition, SACF assay (Fig. 2e) showed that the number of cell colonies in the oeLncRNA DLX6-AS1 group was significantly larger, while that in the shLncRNA DLX6-AS1 group was clearly smaller, suggesting that overexpression of DLX6-AS1 improved amplification of LCSCs. EdU staining used for the detecting cell proliferation shows how the proportion of EdU positive cells in the oeLncRNA DLX6-AS1 group was much higher than that in the blank and NC groups. Besides, the proportion of EdU positive cells in the shLncRNA DLX6-AS1 group was significantly lower compared to the blank and NC groups which highlights cell proliferation was enhanced when DLX6-AS1 was overexpressed (Fig. 2f). All these findings illustrate that down-regulation of DLX6-AS1 could inhibit the self-renewal, amplification, and proliferation of LCSCs.

**Fig. 2:** Reducing lncRNA DLX6-AS1 inhibits self-renewal, amplification, and proliferation of LCSCs. **a**, expression of LCSCs markers at mRNA levels detected by RT-qPCR; **b** and **c**, expression of LCSCs markers at protein levels detected by western blot analysis; **d**, spheroid formation ability of LCSCs detected by Onco-spheroid formation assay, scale bar = 25 μm; **e**, colony formation ability of LCSCs detected by soft agar colony formation (SACF) assay, scar bar = 50 μm; **f**, proliferation of LCSCs detected by EdU staining, scale bar = 50 μm;^*^, *p* < 0.05, vs. the blank group; the statistical data were expressed as mean value of standard error and analyzed by one-way ANOVA; ANOVA, analysis of variance; the experiment was conducted 3 times; RT-qPCR, reverse transcription quantitative polymerase chain reaction; LCSCs, liver cancer stem cells; LncRNA, long non-coding RNA; DLX6-AS1, DLX6 antisense RNA 1; LCSCs, liver cancer stem cells

### Silenced lncRNA DLX6-AS1 inhibits tumorigenesis and tumor growth of LCSCs in vivo

To further elucidate the role of DLX6-AS1 in LCSCs, LDA and tumor xenograft in NOD-SCID mice were conducted in vivo to examine the tumorigenicity and stem cell proportion of LCSCs. LDA showed that the number of tumors and the proportion of tumor stem cells in the oeLncRNA DLX6-AS1 group were significantly higher than those in the blank and NC groups (Table 2 and Fig. 3a). Tumor xenograft in NOD-SCID mice showed that tumors in the oeLncRNA DLX6-AS1 group appeared earlier, grew faster, and exhibited a larger volume, while the tumors in the shLncRNA DLX6-AS1 group showed the opposite results when compared to the blank and NC groups (all *p* < 0.05) (Fig. 3b-d). These results revealed suppressing the tumorigenesis and tumor growth of LCSCs could be achieved by inhibiting lncRNA DLX6-AS1.

**Table 2:** Tumorigenicity of Huh7 spheroid cells

Injected cells	Blank	NC	oeLncRNA DLX6-AS1	shLnRNA DLX6-AS1
1000	0/3	1/3	2/3	0/3
5000	1/3	1/3	2/3	0/3
10,000	2/3	2/3	3/3	1/3
50,000	2/3	2/3	3/3	2/3
Total	5/12	6/12	10/12	3/12

Note: NC, negative control; lncRNA, long non-coding RNA; DLX6-AS1, DLX6 antisense RNA 1

**Fig. 3:** Down-regulating lncRNA DLX6-AS1 suppresses tumorigenesis and tumor growth of LCSCs. **a**, the proportion of LCSCs in mice of different groups determined by LDA; **b**, size of subcutaneous tumors in mice of different groups; **c**, weight of subcutaneous tumors in mice of different groups; **d**, volume of subcutaneous tumors in mice of different groups; *N* = 8; ^*^, *p* < 0.05, vs. the blank group; the statistical data were expressed as mean value of standard error and analyzed by one-way ANOVA; ANOVA, analysis of variance; the experiment was conducted 3 times; LDA, limiting dilution assay; LCSCs, liver cancer stem cells; lncRNA, long non-coding RNA; DLX6-AS1, DLX6 antisense RNA 1

### LncRNA DLX6-AS1 inhibits CADM1 expression by promoting methylation of the CADM1 promoter

DLX6-AS1 was initially predicted to be localized in the nucleus by the lncATLAS website (Fig. 4a), which was confirmed by FISH (Fig. 4b). Sequence blasting identified complementary base pairing between DXL6-AS1 and CADM1 promoter region (Fig. 4c). The MEM website helped further confirm that CADM1 was indeed a target gene of DLX6-AS1 (Fig. 4d). Dual-luciferase reporter gene assay revealed that compared with the NC group, the luciferase activity of cells transfected with CADM1-WT in the oeLncRNA DXL6-AS1 group decreased significantly (*p* < 0.05), while there was no significant change in luciferase activity in cells transfected with CADM1-MUT between the NC and oeLncRNA DXL6-AS1 groups (Fig. 4e). This further highlights how DXL6-AS1 could downregulate the transcription of CADM1. To elucidate the binding of DXL6-AS1 to CADM1 promoter region, CHIP and RIP assays were conducted in LCSCs. As shown in Fig. 4f, the enrichment of methyltransferase DNMT1, DNMT3a, and DNMT3b in the CADM1 promoter region could be observed obviously. Additionally, Fig. 4g shows the oeLncRNA DLX6-AS1 group exhibited a higher conjugation rate with DNMT1, DNMT3a, and DNMT3b (all *p* < 0.05), while the shLncRNA DLX6-AS1 group showed opposite results when compared with the blank group (all *p* < 0.05).

**Fig. 4:** Down-regulating lncRNA DLX6-AS1 increases CADM1 expression via blockade of methylation of the CADM1 gene promoter region. **a**, subcellular localization of lncRNA DLX6-AS1 predicted by lncATLAS website; **b**, subcellular localization of LncRNA DLX6-AS1 detected by FISH, scale bar = 25 μm; **c**, Potential binding sites between LncRNA DLX6-AS1 and CADM1 analyzed by Blast; **d**, prediction of target genes of lncRNA DLX6-AS1 by MEM website; **e**, regulation of CADM1 by LncRNA DLX6-AS1 determined by dual-luciferase reporter gene assay, ^*^, *p* < 0.05, vs. the NC group; **f**, fold enrichment of DNMT1, DNMT3a, and DNMT3b in the CADM1 promoter determined by CHIP-RT-qPCR, ^*^, *p* < 0.05, vs. the Input group; **g**, fold enrichment of DNMT1, DNMT3a, and DNMT3b in the blank, oeLncRNA DXL6-AS1, and shLncRNA DXL6-AS1 groups determined by RIP-RT-qPCR, ^*^, *p* < 0.05, vs. the blank group; **h**, the methylation of CADM1 promoter by BSP (black circle, methylation site; white circle, unmethylation site); **i**, distribution of CpG island in CADM1 gene promoter region; **j**, the methylation of CADM1 promoter detected by MSP (U, Unmethylation; M, methylation); **k-l**, expression of DLX6-AS1 and CADM1 determined by RT-qPCR, ^*^, *p* < 0.05, vs. the blank group; **m-n**, protein levels of CADM1 determined by western blot analysis, ^*^, *p* < 0.05, vs. the blank group; the statistical data were expressed as mean value of standard error, the differences between two groups were analyzed by the *t* test, and others were analyzed by one-way ANOVA; the experiments were conducted 3 times; blast, basic local alignment search tool; CADM1, cell adhesion molecule 1; ANOVA, analysis of variance; RT-qPCR, reverse transcription quantitative polymerase chain reaction; lncRNA, long non-coding RNA; DLX6-AS1, DLX6 antisense RNA 1; FISH, fluorescence in situ hybridization; CHIP, chromatin immunoprecipitation; DNMT1, DNA methyltransferase-1; DNMT3a, DNA methyltransferase-3a; DNMT3b, DNA methyltransferase-3b; BSP, bisulfite sequencing PCR; MSP, methylation specific PCR

Furthermore, the methylation of the CpG sites in the CADM1 promoter region was determined using MSP and BSP in LCSCs (Fig. 4i). The CpG island of CADM1 in the oeLncRNA DXL6-AS1 group was highly methylated and poorly methylated in the shLncRNA DXL6-AS1 group (Fig. 4h, j), suggesting that the methylation of CpG island of CADM1 gene was related to the expression of DXL6-AS1. RT-qPCR and western blot analysis (Fig. 4k-n) suggested that in comparison with the blank group, the oeLnc DXL6-AS1 group displayed a reduction in CADM1 levels, which was opposite to what was found in the shLncRNA DLX6-AS1 group. These findings showed lncRNA DLX6-AS1 was able to downregulate the expression of CADM1 by promoting the methylation of CADM1 promoter region.

### LncRNA DLX6-AS1 downregulation inactivates the STAT3 signaling pathway by upregulating CADM1 in LCSCs

A small molecule inhibitor of STAT3 S3I-201 was employed in order to investigate the role of STAT3 signaling pathway in LCSCs. The nuclear translocation of STAT3 detected by immunofluorescence staining was considered as an indicator that reflects the activation of the STAT3 signaling pathway. The nuclear import of STAT3 in the LCSCs was increased in the shCADM1 group, and decreased in the S3I-201 group, suggesting that knocking down of CADM1 activated the STAT3 signaling pathway (Fig. 5a). Moreover, RT-qPCR and western blot analysis (Fig. 5b-e) detected the phosphorylation of CADM1 and STAT3 and showed that the shCADM1 group exhibited a reduction in mRNA and protein expression of CADM1 as well as higher phosphorylation level of STAT3. This indicated increased STAT3 activity led to STAT3 signaling pathway activation, while the reverse trend was found in the S3I-201 group. These results provided evidence of how lncRNA DLX6-AS1 silencing could inactivate the STAT3 signaling pathway by elevating CADM1 in LCSCs.

**Fig. 5:** Reducing lncRNA DLX6-AS1 suppresses the STAT3 signaling pathway via the upregulation of CADM1. **a**, nuclear import of STAT3 detected by immunofluorescence staining, scale bar = 25 μm; **b**, CADM1 expression in LCSCs isolated from Huh7 and HepG2 determined by RT-qPCR; **c-e**, CADM1 protein levels and phosphorylation levels of STAT3 in LCSCs isolated from Huh7 and HepG2 determined by western blot analysis; ^*^, *p* < 0.05, vs. the blank group; the statistical data were expressed as mean value of standard error and analyzed by one-way ANOVA; the experiment was conducted 3 times; CADM1, cell adhesion molecule 1; STAT3, signal transducer and activator of transcription 3; RT-qPCR, reverse transcription quantitative polymerase chain reaction; ANOVA, analysis of variance; lncRNA, long non-coding RNA; DLX6-AS1, DLX6 antisense RNA 1

### Down-regulation of lncRNA DLX6-AS1 inhibits the spheroid formation ability, colony formation ability, and proliferation ability of LCSCs by increasing CADM1 and suppressing STAT3 signaling pathway

Low-adhesion spheroid formation LCSCs isolated from Huh7 and HepG2 was conducted to explore the effects of lncRNA DLX6-AS1 on LCSCs. In comparison with the blank and NC groups, the shCADM1 group showed significantly higher mRNA and protein expression of CD133, CD13, Nanog, SOX2, and OCT-4 (Fig. 6a-c), and upregulated spheroid formation ability, colony formation ability, and proliferation ability of LCSCs (Fig. 6d-f). This contrasts to that of the S3I-201 group, which showed the opposite results which inhibited the STAT3 signaling pathway. However, mRNA and protein levels of CD133, CD13, Nanog, SOX2, and OCT-4, spheroid formation ability, colony formation ability, and proliferation ability did not differ among the oeLncRNA DLX6-AS1 + shCADM1, shCADM1 + S3I-201, blank, and NC groups. These results suggested downregulation of lncRNA DLX6-AS1 could lead to suppressed spheroid formation ability, colony formation ability, and proliferation ability of LCSCs through inactivating the STAT3 signaling pathway by upregulating CADM1.

**Fig. 6:** Reduced lncRNA DLX6-AS1 inhibits spheroid formation ability, colony formation ability, and proliferation ability of LCSCs via the inhibition of CADM1–mediated STAT3 signaling pathway. **a**, mRNA levels of LCSCs markers determined by RT-qPCR; **b** and **c**, protein levels of LCSCs markers determined by western blot analysis; **d**, spheroid formation ability of LCSCs detected by spheroid formation assay, scale bar = 100 μm; **e**, colony formation ability of LCSCs detected by colony formation assay, scar bar = 50 μm; **f**, proliferation ability of LCSCs determined by EdU staining, scale bar = 50 μm; ^*^, *p* < 0.05, vs. the blank group; the statistical data were expressed as mean value of standard error and analyzed by one-way ANOVA; the experiment was conducted 3 times; CADM1, cell adhesion molecule 1; STAT3, signal transducer and activator of transcription 3; RT-qPCR, reverse transcription quantitative polymerase chain reaction; ANOVA, analysis of variance; LCSCs, liver cancer stem cells; lncRNA, long non-coding RNA; DLX6-AS1, DLX6 antisense RNA 1; CD133, prominin-1; CD13, aminopeptidase N

### Downregulated lncRNA DLX6-AS1 suppresses tumorigenesis and tumor progression in vivo via inactivation of the CADM1-dependent STAT3 signaling pathway

The LDA (Table 3 and Fig. 7a) was conducted for the purpose of exploring the roles of lncRNA DLX6-AS1 and STAT3 signaling pathway in tumor growth in vivo. Results showed that that in contrast to the blank and NC groups, the shCADM1 group exhibited an increase in the number of tumors and proportion of tumor stem cells, while the S3I-201 group showed opposite results. In addition, tumor xenograft in NOD-SCID mice was also conducted, and results demonstrated that compared with the blank and NC groups, tumors in the shCADM1 group developed earlier, grew faster and larger, while those in the S3I-201 group showed the reverse trend; The formation time, growth speed, and tumor size did not significantly differ among the oeLncRNA DLX6-AS1 + shCADM1, shCADM1 + S3I-201, blank, and NC groups (Fig. 7b-d). These results highlighted the inhibition of lncRNA DLX6-AS1 could suppress tumorigenesis and tumor growth of LCSCs in vivo by suppressing the STAT3 signaling pathway after increasing CADM1.

**Table 3:** Tumorigenicity of Huh7 spheroid cells

Injected cells	Blank	NC	shCADM1	S3I-201	shLncRNA DLX6-AS1 + shCADM1	shCADM1 + S3I-201
1000	0/3	0/3	2/3	0/3	0/3	0/3
5000	1/3	1/3	3/3	0/3	1/3	1/3
10,000	1/3	1/3	3/3	1/3	2/3	1/3
50,000	2/3	2/3	3/3	1/3	2/3	2/3
Total	4/12	4/12	11/12	2/12	5/12	4/12

Note: NC, negative control; CADM1, cell adhesion molecule 1; lncRNA, long non-coding RNA; DLX6-AS1, DLX6 antisense RNA 1

**Fig. 7:** Decreased lncRNA DLX6-AS1 represses tumorigenicity and progression of tumors of LCSCs in vivo through inhibiting the activation of the STAT3 signaling pathway by up-regulating CADM1. **a**, proportion of stem cells in mice of 6 groups determined by LDA; **b**, size of subcutaneous tumor in mice of 6 groups detected by tumor xenograft in NOD-SCID mice; **c**, mass of subcutaneous tumor in mice of 6 groups; **d**, volume of subcutaneous tumor in mice of 6 groups; *N* = 8; ^*^, *p* < 0.05, vs. the blank group; the statistical data were expressed as mean value of standard error and analyzed by one-way ANOVA; the experiment was conducted 3 times; ANOVA, analysis of variance; CADM1, cell adhesion molecule 1; STAT3, signal transducer and activator of transcription 3; LDA, limiting dilution assay; LCSCs, liver cancer stem cells; lncRNA, long non-coding RNA; DLX6-AS1, DLX6 antisense RNA 1

## Discussion

HCC is well recognized malignant tumor worldwide, which is characterized by high malignancy, a high risk of metastasis, as well as high occurrence and recurrence rates [22]. Current standard treatment approaches for treating patients with HCC remain unsatisfactory due to poor prognosis rates despite early detection. Therefore, more potential therapeutic targets are required to improve HCC patient’s outcome and mortality [23]. It has been proved that lncRNAs are implicated in the genesis and development of many tumors [24]. In the present study, we aimed to shed light on the potential mechanism of how lncRNA DLX6-AS1 affects tumorigenesis and development of LCSCs. Our findings provided evidence demonstrating that lncRNA DLX6-AS1 silencing could lead to reduced methylation of CADM1 promoter, which further enhanced the expression of CADM1 and inactivated the STAT3 signaling pathway, thus repressing the tumorigenicity and tumor progression of LCSCs.

Initially, we found that lncRNA DLX6-AS1 was up-regulated in HCC tissues, and that down-regulation of lncRNA DLX6-AS1 could contribute to repressed self-renewal, amplification, and proliferation of LCSCs. The crucial role of lncRNA DLX6-AS1 in the tumor progression of HCC has been widely reported, and that abnormal overexpression of lncRNA DLX6-AS1 could be correlated to poor prognosis in patients suffering from HCC [12], which were consistent with our findings. Additionally, lncRNA DLX6-AS1 overexpression has also been found in other carcinomas such as renal cell carcinoma (RCC) and lung adenocarcinoma, serving a pivotal part in cancer development [25]. Abnormal expression of lncRNA DLX6-AS1 in lung adenocarcinoma was demonstrated to be related to the tumor-node-metastasis (TNM) stage and histological differentiation [26]. Taken together, extensive amount evidence has shed a lot of light on how inhibiting lncRNA DLX6-AS1 could lead to a reduction in tumorigenesis and cancer development of HCC by inhibiting the self-renewal, amplification, and proliferation of LCSCs.

The present study also demonstrated that higher methylation levels at the CADM1 promoter region and lower CADM1 expression were both presented in LCSCs. CADM1, a member belonging to the immunoglobulin superfamily of cell adhesion molecule, is an extensively known tumor suppressor [27]. DNA methylation is a physiological process by which methyl groups are added to DNA molecules. In pathological conditions such as cancer, DNA hypermethylation can result in increased tumorigenicity [28, 29]. High methylation of the CADM1 promoter was reported in several cancers such as cervical carcinomas, cell lung carcinoma and pancreatic cancers [30–32]. On the other hand, CADM1 downregulation induced by promoter methylation has been suggested to be important for the pathogenesis of HCC [16], which is largely in agreement with the observations of our study. Our study strongly suggests that upregulation of lncRNA DLX6-AS1 was able to lead to a reduction in CADM1 expression by increasing CADM1 methylation, thus activating the STAT3 signaling pathway. STAT3 is a potent modulator of tumorigenesis, survival, and inflammation of liver cells, is constitutively activated in the vast majority of HCC cells [23]. It has been demonstrated by a recent study that STAT3 is implicated in regulating microenvironment and development of cancers [33]. In accordance with our study, CADM1 has been identified to exhibit a suppressive effect on STAT3 in patients with SqCC [18]. Han et al. suggested that inhibition of STAT3 signaling pathway was able to regulate tumor growth in HCC patients by inhibiting cell proliferation yet inducing cell apoptosis [34]. S31–201, an inhibitor of the STAT3 signaling pathway, has been demonstrated to have an inhibitory effect on cell growth in HCC [35]. STAT3 signaling pathway plays an important role in a variety of CSCs, including breast cancer stem cells [36, 37], LCSCs [38, 39], pancreatic cancer stem cells [40], ovarian cancer stem cells [41], and regulates many downstream pluripotent genes-related to CSCs including OCT4, SOX2, and Nanog [42]. Interestingly, STAT3 was also reported to be a critical factor or a promoter in the expansion of LCSCs promoted by lncARSR [43]. Our findings proved that silencing of lncRNA DLX6-AS1 enforced the expression of CADM1 and inactivated the STAT3 signaling pathway by suppressing CADM1 promoter methylation, thus repressing the tumorigenesis and tumor progression of LCSCs.

## Conclusion

In summary, our results suggested that lncRNA DLX6-AS1 could serve as an oncogene in LCSCs by which silenced DLX6-AS1 contributes to decrease of the methylation of CADM1 promoter and inactivation of the STAT3 signaling pathway, thus exerting suppressive effects on tumorigenesis and tumor development of LCSCs (Fig. 8). Therefore, lncRNA DLX6-AS1 may serve as a novel biomarker for the treatment of HCC.

**Fig. 8:** The molecular mechanism involved in lncRNA DLX6-AS1 affecting LCSCs by regulating STAT3 signaling pathway through affecting CADM1 promoter methylation. Down-regulation of lncRNA DLX6-AS1 inhibited CADM1 promoter methylation, increased CADM1 expression, and suppressed the activation of the STAT3 signaling pathway, and finally the expression of CD133 and CD13 in LCSCs were decreased and the progression of LCSCs was repressed. lncRNA DLX6-AS1, long non-coding RNA DLX6-AS1; CADM1, cell adhesion molecule; STAT3, signal transducer and activator of transcription 3; LCSC, liver cancer stem cells

## Additional file

Additional file 1: **Table S1.** Correlation between DLX6-AS1 expression and clinicopathological characteristic of HCC patients. (DOCX 16 kb)

## Data Availability

The datasets generated/analyzed during the current study are available.

## Abbreviations

CADM1: Cell adhesion molecule 1
cDNA: Complementary DNA
ChIP: Chromatin immunoprecipitation
DEGs: Differentially expressed genes
DLX6-AS1: Distal-less homeobox 6 antisense 1
DMEM: Dulbecco’s modified Eagles Medium
DNMT: DNA methyltransferase
ELDA: Extreme limiting dilution analysis
FDR: False positive discovery
FGF: Fibroblast growth factors
FISH: Fluorescence in situ hybridization
GAPDH: Glyceraldehyde-3-phosphate dehydrogenase
HBV/HCV: Hepatitis B/C virus infections
HCC: Hepatocellular carcinoma
IgG: Immunoglobulin G
KEGG: Kyoto Encyclopedia of Genes and Genomes
LAC: Lung adenocarcinoma
LCSCs: Liver cancer stem cells
LDA: Limiting dilution assay
lncRNAs: Log non-coding RNAs
MSP: Methylation specific PCR
MUT: Mutant type
NC: Negative control
OS: Overall survival
PBST: Phosphate-Buffered Saline with Tween 20
PVDF: Polyvinylidene fluoride
RCC: Renal cell carcinoma
RIP: RNA immunoprecipitation
RIPA: Radioimmunoprecipitation
RT-qPCR: Reverse transcription quantitative polymerase chain reaction
SACF: Soft agar colony formation
SDS: Sodium dodecyl sulfate
SDS-PAGE: Sodium dodecyl sulfate-polyacrylamide gel electrophoresis
SqCC: Squamous cell carcinomas
STAT3: Signal transducer and activator of transcription 3
TCGA: The Cancer Genome Atlas
TNM: Tumor-node-metastasis
WT: Wild-type
